# miR-337-5p promotes the development of cardiac hypertrophy by targeting Ubiquilin-1 (UBQLN1)

**DOI:** 10.1080/21655979.2021.1964892

**Published:** 2021-09-13

**Authors:** Ying Ding, Jingyu Wang, Jun Lu

**Affiliations:** Electrocardiographic Function Department, Xiangyang Central Hospital, Affiliated Hospital Of Hubei University Of Arts And Science, Xiangyang, Hubei, China

**Keywords:** miR-337-5p, UBQLN1, cardiac hypertrophy, mTOR, p70S6K

## Abstract

Cardiac hypertrophy is an adaptive response of the myocardium to the pressure overload of the heart. MicroRNAs (miRNAs/miRs) are shown to be directly involved in the development of cardiac hypertrophy. However, the function of miR-337-5p and its potential contribution to the serine/threonine-protein kinase, a mammalian target of rapamycin (mTOR) signaling in cardiac hypertrophy remains unknown. In the present study, miR-337-5p expression was examined in cardiomyocytes treated with angiotensin II (Ang II). An adenovirus vector system was employed to knockdown miR-337-5p expression to investigate its functions in cardiac hypertrophy. The results revealed a significant increase in the expression of miR-337-5p in cardiomyocytes treated with Ang II as compared with controls. In addition, downregulation of miR-337-5p expression inhibited cardiac hypertrophy both *in vitro* and *in vivo*. Dual-luciferase reporter assays demonstrated Ubiquilin-1 (*UBQLN1)* as the direct target of miR-337-5p, and revealed its function in the modulation of mTOR signaling. Rescue experiments indicated that *UBQLN1* overexpression reversed the effects of miR-337-5p, and further verified this interaction. In summary, the results of the present study show that miR-337-5p silencing attenuates cardiac hypertrophy by targeting *UBQLN1*. Therefore, miR-337-5p plays a critical role in cardiac hypertrophy and may serve as a new therapeutic target.

## Introduction

Cardiac hypertrophy is an adaptive response of the myocardium to the pressure overload of the heart. This phenomenon results in the enlargement of the heart muscle and correspondingly decreases the size of the chambers of the heart [1,2]. Cardiac hypertrophy is a critical determinant for the progression of heart failure and is closely related to a high risk of sudden cardiac death [3]. Diverse pathological stimuli such as myocardial infarction, hypertension, valvular insufficiency, and mutations of contractile proteins contribute to the development of cardiac hypertrophy [4]. The process of cardiac hypertrophy is characterized with the pathological remodeling of the ventricles, and may be accompanied with an increase in the size of cardiomyocytes without any alteration in cardiomyocyte number [5]. The increase in the muscle mass is accompanied with enlargement of myocytes in response to various pathophysiological insults, including angiotensin II (Ang II). A series of simultaneous alterations in both intracellular signaling pathways and expression of transcriptional mediators in cardiomyocytes guides protein synthesis and directs a phenotype shift [6].

MicroRNAs (miRNAs) are a group of endogenous noncoding single-stranded small molecule RNAs comprising 21–23 nucleotides. miRNAs are found in many organisms and regulate gene expression at the post-transcriptional level by binding to the 3ʹ-untranslated regions (3ʹ-UTRs) of target mRNAs. Recent functional studies have demonstrated the application of both gain- and loss-of-function approaches in mice to uncover the important roles of miRNAs in cardiac hypertrophy and ventricular remodeling [7,8].

It is becoming increasingly apparent that various miRNAs are directly involved in the development of cardiac hypertrophy, including miR-206 [9], miR-451 [10], miR-21 [11], miR-155 [12], and miR-22 [13]. Genetic studies have revealed that miR-337-5p participates in solid tumor progression [14], hematological malignancy, and several ischemia-related diseases [15]. miR-337-5p was also found to be dysregulated in chronic doxorubicin treatment-induced heart failure [16]. Microarray analysis in a heart failure mouse model revealed the upregulation in miR-337-5p expression in the heart at 5 and 28 days after model initiation [16].

Ubiquilin-1 (UBQLN1) is a key adaptor protein that is thought to play a role in the endoplasmic reticulum and ubiquitin-proteasome system for protein degradation. UBQLN1 is known to alter autophagic activity in the lysosome and is related to aggregation of misfolded proteins, cellular dysfunction, and diseases. This mechanism has been linked to several disorders, including Alzheimer’s disease, spinocerebellar ataxia type 1, Huntington’s disease, and cancer [17].

We have previously examined the expression of miR-337-5p in cardiac hypertrophy, and demonstrated its expression upregulation in Ang II–induced cardiac hypertrophy. We speculate that miR-337-5p plays critical roles in the progression of cardiac hypertropy. In the present study, we aim to investigat its potential regulation and the possible contribution of its predicted target UBQLN1 and the related mTOR signaling pathway to cardiac hypertrophy progression.

## Materials and methods

### Animals and experimental procedures

All animal procedures were approved by the Animal Research Committee of Affiliated Hospital Of Hubei University of Arts and Science according to the Guide for the Care and Use of Laboratory Animals published by the United States National Institutes of Health. C57BL/6 mice (n = 60, age, 8 weeks; weight, 25–30 g) were obtained from Beijing Vital River Laboratory Animal Center and maintained in the animal facility for 1 week before surgery. After intraperitoneal injection with 1% pentobarbital (50 mg/kg), the aorta was ligated with a 7–0 silk thread placed around the vessel using a 26-gauge needle to ensure consistent occlusion. Mice from the sham group underwent the same surgery without thread ligation. Mice were transduced with ad-sh-miR-337-5p (anti-miR: 5ʹAACTCCTGTATGTTGCCGTTC3ʹ) and ad-sh-NC (anti-NC:5ʹAATTCGAAGCCGATCGGCGTACT’) (3.5 × 10^7^ viral particles/mouse, GenePharma Co., Ltd, China) via injection into the heart 1 week after TAC. After 4 weeks, the mice were euthanized by injection of an excess of pentobarbital. Their hearts were collected, and the left ventricles were rapidly frozen in liquid nitrogen and stored at −80°C for subsequent experiments (18. 19).

### Primary cultures of neonatal mouse cardiomyocytes and transfections

Neonatal mouse cardiomyocytes were isolated from the hearts of newborn C57BL6 mice (1-day-old). The hearts were quickly excised, and the ventricles were transferred into cold Hank’s balanced salt solution without Ca^2+^ and Mg^2+^ (Invitrogen, Thermo Fisher Scientific, Inc). Cells were detached from the ventricle tissue. Isolated cardiomyocytes were cultured in Dulbecco’s modified Eagle’s medium (Gibco, Thermo Fisher Scientific, Inc) containing 10% fetal bovine serum (Gibco, Thermo Fisher Scientific, Inc) supplemented with antibiotics (penicillin, streptomycin; Gibco, Thermo Fisher Scientific, Inc). Cells were maintained at 37°C under humidified conditions of 95% air and 5% CO_2_. The cardiomyocytes were cultured in a semi-confluent condition to prevent cellular differentiation. The cells were plated in a six-well plate at a density of 2 × 10^5^ cells/well. After 24 h of culture, the cells were transduced with ad-sh-NC or ad-sh-miR-337-5p at 2 × 10^5^ viral particles/mL. After 12 h, the culture medium was replaced with serum-free medium, and the cells were incubated for additional 48 h in the presence or absence of 1 μM Ang II (Sigma-Aldrich; Merck KGaA) [19].

### RNA isolation and reverse-transcription quantitative polymerase chain reaction (RT-qPCR)

Total RNA from the heart or cardiomyocytes was extracted using Trizol Reagent (Invitrogen, Thermo Fisher Scientific, Inc), following the manufacturer’s instructions. For reverse transcription, 600 ng of total RNA was used with SuperScript II RNase H Reverse Transcriptase kit (Invitrogen, Thermo Fisher Scientific, Inc) according to the manufacturer’s protocol. qPCR was performed using the SYBR Green PCR master mix (Invitrogen, Thermo Fisher Scientific, Inc), and the mRNA levels of target genes were normalized to glyceraldehyde 3-phosphate dehydrogenase (*GAPDH*) gene expression level. The level of miR was normalized to U6. Relative expression was evaluated by the 2^–ΔΔCt^ method. All experiments were independently performed in triplicates. The primers used are as follows: forward CACAGATCTGATGGATTTCAAGA and reverse:CCTCATCTTCTACCGGCATC for atrialnatriureticpeptide (ANP); forward: GTCAGTCGTTTGGGCTGTAAC and AGACCCAGGCAGAGTCAGAA for Brain natriuretic peptide (BNP); forward:CCGAGTCCCAGGTCAACAA and reverse:CTTCACGGGCACCCTTGGA for β-myosin heavy chain (β-MHC). forward:ATCCATAGCAGCGGATCGACT and reverse:CAGGATAGCATGCAGACTTAGC for miR-337-5p; forward:ACTCCACTCACGGCAAATTC and reverse:TCTCCATGGTGGTGAAGACA for GAPDH. Forward: CACAGATCTGATGGATTTCAAGA and reverse:CCTCATCTTCTACCGGCATC for U6 [19].

### 3ʹ-UTR luciferase reporter assays

293 T cells were transfected with the full-length 3ʹ-UTR of *UBQLN1* downstream of the *Renilla* luciferase gene in the presence of either miR-337-5p mimic or control miRNA mimic and co-transfected with a pGL3-basic control plasmid (firefly luciferase, Promega Corporation) to generate pGL3-basic- UBQLN1-3ʹ-UTR-wild type (WT: GGGTGAAAAACAAAGAGCCGTTT). A seed sequence transversion (mutated version of the UBQLN1 3ʹ-UTR), named pGL3-basic-UBQLN1-3ʹ-UTR-Mutant (mut: GGGTGAAAAACAAAGAGGGCATT), was constructed as a control. After 24 h after transfection, the cell lysates were collected and sequentially used for the detection of luciferase activity. Relative firefly luciferase activity, which was normalized to *Renilla* luciferase activity, was measured using a dual luciferase reporter gene assay system (Promega, Corporation) according to the manufacturer’s instructions. All experiments were independently performed in triplicates [19].

### Western blot analysis

Cells were lysed in ice-cold radioimmunoprecipitation assay (RIPA) lysis buffer containing ethylenediaminetetraacetic acid (EDTA)-free protease inhibitor cocktail (Roche) for 30 min and then centrifuged to remove the Triton-insoluble pellet. Samples normalized with equal protein concentration were subjected to sodium dodecyl sulfate polyacrylamide gel electrophoresis (SDS-PAGE) and western blot analysis. Polyvinylidene fluoride (PVDF) membranes were incubated with the following primary antibodies for overnight at 4°C: UBQLN1 (Abcam, 1:2000), p-mTOR (Abcam, 1:2000), mTOR (Abcam, 1:2000), p-p70S6K (Abcam, 1:2000), p70S6K (Abcam, 1:2000), GAPDH (Sigma, 1:1000). Goat anti-mouse (1:5000) or anti-rabbit (1:5000) secondary antibodies (BBI Life Science Corp.) were used. The protein bands were visualized using chemiluminescence imaging system V1.8.0.112 (Tannon Science & Technology Co., Ltd,). All experiments were independently performed in triplicates [19].

### Immunofluorescence

Cells were fixed in 4% paraformaldehyde and permeabilized with 0.2% Triton X-100 in phosphate-buffered saline (PBS) for 15 min. The cells were then incubated with 5% normal serum that matched the species used to generate the secondary antibody and then probed with α-actin (Abcam, 1:800) primary antibody for overnight at 4°C. The cells were then incubated in fluorochrome-conjugated secondary antibodies for 2 h at room temperature. Cell nucleus was stained with 4ʹ,6-diamidino-2-phenylindole (DAPI; Sigma-Aldrich, Merck KGaA). Images were captured with a Carl Zeiss Axioskop microscope (Carl Zeiss AG, Oberkochen, Germany). The cardiomyocyte diameter was calculated by ImageJ software [19].

### Echocardiography for mice

Echocardiography of the left ventricles of mice 4 weeks after TAC was performed using the Vevo 2100 Imaging System (FUJIFILM, VisualSonics Inc.). Briefly, mice were anesthetized with 2% isoflurane and then maintained under 1.5% isoflurane anesthesia. Each mouse was placed on an examination board with the chest facing up, and all hair in the area of interest was wiped away. A 7.5 MHz probe was used and the M-mode measurements of left ventricular (LV) dimensions conducted using the scan head were calculated from more than three heart cycles. LV inner diameters during diastole and systole were determined from the M-modes along with the heart rate. Diastolic and systolic volumes were obtained by applying Simpson’s rule of discs to serially acquired short axis images. Stroke volume was calculated using the following method: Stroke volume = diastolic volume-systolic volume. Ejection fraction was calculated as follows: ejection fraction = (stroke volume/diastolic volume) × 100%. Cardiac output was determined using the following equation: Cardiac output = stroke volume × heart rate. A total of six C57BL/6 mice from each group were tested [20].

### Histological analysis

Mouse heart tissues were collected 4 weeks after TAC. The heart was fixed with paraformaldehyde, embedded in paraffin and cut into slices of 4 μm thickness for histological analysis. The size and morphological alterations of the heart tissue were assessed by hematoxylin/eosin (HE) and Masson trichrome staining. Paraffin-embedded tissue sections were stained with mouse monoclonal α-sarcomeric actin (α-actin) antibody (1:75, Abcam) and Alexa Fluor 594 goat anti-mouse antibody (1:200, Abcam) as secondary antibody. Cell nucleus was stained with DAPI (Sigma-Aldrich, Merck KGaA). Sections were mounted and analyzed under a confocal microscope (Zeiss, GmbH). The heart tissues collected from six mice in each group were analyzed [20].

### Bioinformatics analysis

TargetScan Mouse Release 7.2 was run on input lists to find predicted miR-337-5p binding sites [21].

### Statistical analysis

All data are presented as the mean ± standard deviation (SD). Statistical analyses were performed using one-way analysis of variance (ANOVA) and Student’s test. The data were analyzed using GraphPad Prism 5.0, and p < 0.05 was considered to be statistically significant. All experiments were independently performed triplicates.

## Results

MiR-337-5p was found up-regulated in cardiac hypertrophy. We speculate that miR-337-5p plays critical roles in the progression of cardiac hypertropy. In the present study, we aim to investigat its potential regulation and the possible contribution of its predicted target UBQLN1 and the related mTOR signaling pathway to cardiac hypertrophy progression. The in vitro and in vivo model of cardiac hypertrophy were established to evaluate the effect of miR-375-5p on the cardiac hypertrophy. Luciferase and RNA pull down assay were performed to investigate the interaction between miR-375-5p and UBQLN1. The downstream signaling pathway mTOR/p70S6K was also explored.

### Expression of miR-337-5p is upregulated in cardiac hypertrophy

To analyze the expression pattern of miR-337-5p in cardiac hypertrophy, an *in vitro* hypertrophic model was established by treating cardiomyocytes with Ang II. The immunofluorescence staining of α-actin indicated that Ang II-treated cardiomyocytes had a larger size than the control cells (Figure 1(a)). The expression levels of ANP, BNP, and β-MHC markedly increased in hypertrophic cardiomyocytes as compared with those in control cells by using qPCR evaluation (Figure 1(b,c)). We evaluated the expression of miR-375-5p in the cardiomyocytes under Ang II treatment. qPCR results revealed the significant upregulation in the expression of miR-337-5p in cardiomyocytes treated with Ang II as compared with that in the control cells (Figure 1(d)). This result indicates that miR-337-5p may participate in the pathogenesis of cardiac hypertrophy.

**Figure 1.** miR-337-5p expression is upregulated in cardiomyocytes subjected to Ang II treatment. (a) The morphology and size of cardiomyocytes subjected to Ang II treatment were evaluated by immunofluorescence staining of α-actin (n = 6). (b, c) The levels of myocardial hypertrophy biomarkers ANP, BNP, and β-MHC were detected using qPCR (n = 3). (d) The expression of miR-337-5p was detected with qPCR (n = 3). **p < 0.01

### miR-337-5p aggravates cardiac hypertrophy in vitro

To confirm the role of miR-337-5p in cardiac hypertrophy, adenovirus-mediated silencing of miR-337-5p (anti-miR) expression was performed. As expected, the relative level of miR-337-5p sharply decreased in cardiomyocytes after the transduction of anti-miR as compared with that in the cells treated with control adenovirus (anti-NC) (Figure 2(a)). The qPCR results indicated that inhibition of miRNA-337-5p expression led to a significant decrease in the expression levels of ANP, BNP, and β-MHC as well as the size of the cardiomyocyte as compared with the anti-NC treatment group (Figure 2(b,c)).

**Figure 2.** miR-337-5p expression knockdown ameliorates the Ang II–induced cardiomyocyte hypertrophy. (a) miR-337-5p expression was downregulated in cardiomyocytes subjected to anti-miR-337-5p treatment (n = 3). (b) The morphology and size of cardiomyocyte were detected by immunofluorescence staining of α-actin (n = 6). (c) The levels of myocardial hypertrophy biomarkers ANP, BNP, and β-MHC were detected using qPCR (n = 3). **p < 0.01

### miR-337-5p induces cardiac hypertrophy by targeting UBQLN1 and activating the mTOR signaling pathway

To explore the mechanism underlying miR-337-5p activity in cardiac hypertrophy, the potential target genes of miR-337-5p were investigated using bioinformatic analysis. The 3ʹ-UTR of *UBQLN1* gene was found to contain a highly conserved miR-337-5p seed sequence, suggesting that *UBQLN1* may be a target of miR-337-5p (Figure 3(a)). To validate this prediction, wild-type and mutant sequences of *UBQLN1* were separately cloned into a luciferase reporter (Figure 3(b)). The luciferase activity of the reporter carrying the WT *UBQLN1* reduced in the presence of miR-337-5p but that of the reporter carrying the mutant *UBQLN1* did not change (Figure 3(c)). To further confirm the relationship between miR-337-5p and UBQLN1, the expression of UBQLN1 in hypertrophic cardiomyocytes was validated. miR-337-5p notably inhibited the mRNA and protein expression of UBQLN1, and miR-337-5p inhibition increased the expression level of UBQLN1 (Figure 3(d-f)). Together, these data indicate that UBQLN1 is a direct target of miR-337-5p.

**Figure 3.** miR-337-5p directly targets UBQLN1 in cardiomyocytes. (a, b) The wild-type and mutant binding sites of miR-337-5p at the 3ʹ-UTR of *UBQLN1* are shown. (c) Luciferase activity assay was performed to identify whether *UBQLN1* is the direct target gene of miR-337-5p. (d) qPCR was performed to evaluate *UBQLN1* expression. (e, f) Western blot analysis was conducted to evaluate the protein expression of UBQLN1 (n = 3). **p < 0.01

### miR-337-5p targets UBQLN1 and activates the mTOR signaling pathway

UBQLN1 specifically binds to mTOR in mammalian cells. Here, we investigated the expression of mTOR in hypertrophic cardiomyocytes using western blot analysis and found that the expression and phosphorylation of mTOR as well as the phosphorylation of p70S6K were upregulated in response to cardiac hypertrophy. Moreover, after the knockdown of miR-337-5p expression, the expression and phosphorylation of mTOR and the phosphorylation of p70S6K reversely declined (Figure 4(a,b)).

**Figure 4.** miR-337-5p regulates the expression of UBQLN1 and the downstream proteins. (a, b) Western blot assay was carried out to evaluate the expression levels of UBQLN1, mTOR, p-mTOR, p70s6k, and p-p70s6k (n = 3). *p < 0.05, **p < 0.01

### Knockdown of UBQLN1 expression reverses the effect of miR-375-5p silencing on cardiac hypertrophy

Rescue experiments were performed to elucidate the role of UBQLN1 in cardiac hypertrophy. First, the expression of UBQLN1 in cultured cardiomyocytes was evaluated by qPCR. The results indicated that the transfection of si-UBQLN1 significantly reduced the expression level of UBQLN1 (Figure 5(a)). Quantification of cardiomyocyte size and expression of hypertrophic genes using immunofluorescence staining of α-actin and western blot, respectively, demonstrated that UBQLN1 knockdown reversed the protective effect of miR-337-5p silencing on cardiac hypertrophy *in vitro* (Figure 5(c,d)).

**Figure 5.** UBQLN1 knockdown reverses the effect of miR-337-5p silencing on cardiomyocyte hypertrophy. (a) The expression level of UBQLN1 was evaluated by qPCR (n = 3). (b) The morphology and size of cardiomyocyte were evaluated by immunofluorescence staining of α-actin (n = 3). (c) The levels of myocardial hypertrophy biomarkers ANP, BNP, and β-MHC were detected using qPCR (n = 3). **p < 0.01

### miR-337-5p aggravates cardiac hypertrophy in vivo

To explore the effect of miR-337-5p on an animal model of cardiac hypertrophy, mice that had been subjected to TAC surgery were injected with anti-miR-337-5p after 1 week of operation. The inhibition of miRNA-337-5p expression led to a decrease in the size of the heart and the ratio of heart weight to tibial length (HW/TL) as compared with control treatment (Figure 6(a,b)). The results of echocardiography indicated that the knockdown of miR-337-5p expression elevated the cardiac function, as evident from left ventricular ejection fraction (LVEF) and left ventricular fractional shortening (LVFS) analysis results, and reduced left ventricular end-diastolic dimension (LVEDd) and left ventricular end-systolic dimension (LVESd) (Figure 6(c)). Taken together, miR-337-5p expression inhibition appears to reduce cardiac hypertrophy both *in vitro* and *in vivo*.

**Figure 6.** miR-337-5p silencing inhibits cardiac hypertrophy *in vivo*. (a) HE staining of the heart tissue was performed to analyze cardiac hypertrophy. (b) The ratio of heart weight to tibial length (HW/TL) was calculated. (c) Cardiac function was evaluated by assessing LVEF, LVFS, LVEDd, and LVESd. **p < 0.01

## Discussion

miRNAs are involved in complex pathological processes by regulating cellular activities. As miR-337-5p was identified as a novel miRNA, most studies have investigated its functional roles in cancer. For instance, miR-337-5p regulates hepatocellular carcinoma cell proliferation, migration, and invasion, and its expression significantly correlates with clinicopathological features and survival outcomes [22,23]. Gastric cancer and pancreatic ductal adenocarcinoma patients with low miR-337-5p levels have worse prognosis than those with high miR-337-5p levels, and miR-337-5p is positively correlated with TNM stage and lymph node status [24]. In addition, miR-337-5p-3p promotes chondrocyte proliferation and reduces ischemic brain injury.

To the best of our knowledge, the role of miR-337-5p-3p in the pathogenesis of cardiovascular diseases remains unknown. The present study demonstrates that miR-337-5p inhibition elevated the cardiac function of mice subjected to TAC surgery and reduced the volume of cardiomyocytes under Ang II treatment. miRNAs bind to and suppress the levels of mRNAs, and consequently influence various biological processes. miR-337-5p has been shown to directly bind to the transcriptional coactivator YAP1 [25,26], transport protein SEC23A [27,28], short stature homeobox protein SHOX2 [29], and ubiquitin-protein ligase E3A [30], and attenuate their expression. The present study focused on UBQLN1, which was predicted to be a potential target of miR-337-5p by bioinformatic analysis. Luciferase reporter assay and rescue experiments confirmed this prediction.

Ubiquilin proteins are structurally conserved and contain a ubiquitin-like domain (UBL) at their N-termini and a ubiquitin-associated domain (UBA) at their C-termini. UBQLN1 is located on chromosome 9q22 and encodes two major isoforms containing either 589 or 561 amino acids, which are adaptors thought to link ubiquitinated proteins to the proteasome [31,32]. Functionally, UBQLN1 binds numerous cytosolic or transmembrane proteins via functional domains and modulates their steady state levels. The functional form of UBQLN1 is not clear, as it is capable of forming homodimers. Evidence suggests that UBQLN1 functions as an adaptor protein that links the ubiquitination machinery to the proteasome and affects protein degradation [33]. Thus, UBQLN1 has been implicated in several physiological and pathological process, including cancer progression [34], neurodegenerative disorders [35], endoplasmic reticulum-associated degradation [36], autophagy [37,38], apoptosis, and receptor trafficking [39]. Most studies on UBQLN1 have focused on its function in neurodegenerative diseases. Investigation of its role in the cardiovascular system revealed that UBQLN1 colocalizes with the proteasome in cardiomyocytes and significantly increases in the soluble fraction following ischemia/reperfusion (I/R) stress [40]. Further research showed that UBQLN1 deletion promoted I/R-induced LV dysfunction and increased the infarct size in mice. These findings indicate the critical role of UBQLN1 in the progression of heart diseases [41].

To clarify the effect of UBQLN1 in cardiac hypertrophy, its expression was knocked down and the subsequent effects on the cardiac function were investigated. The effects of decreased UBQLN1 levels were consistent with the role of miR-337-5p expression. It reversed the effect of Ang II and TAC on cardiomyocytes and the mouse heart. Several studies have identified mTOR as a key regulator of cardiac hypertrophy; for instance, the mTOR inhibitor rapamycin prevented heart-weight gain in an overload model of hypertrophy [5] and blocked cardiomyocyte size increase induced by Ang II [6] and phenylephrine [7] likely by inhibiting protein synthesis [7]. mTOR is a conserved serine/threonine kinase with a key regulatory function in cardiovascular physiology and pathology8 [41–45].

UBQLN1 was reported to specifically bind to a non-catalytic region of the mTOR kinase [46,47]. In the present study, the knockdown of UBQLN1 expression promoted mTOR expression and p70S6K phosphorylation. It can be hypothesized that UBQLN1 regulates the expression of mTOR and the phosphorylation of p70S6K, which play a critical role in the regulation of cardiac hypertrophy. Whether miR-337-5p knockdown can directly decrease the level of mTOR through UBQLN1 will be the focus of our further study.

## Conclusion

In the present study, we found that miR-337-5p knockdown could inhibited cardiac hypertrophy both in vitro and in vivo. It was found to target UBQLN1 and regulate the mTOR/p70S6K signaling. MiR-337-5p plays a critical role in cardiac hypertrophy and may serve as a potential therapeutic target for hypertrophic heart diseases.

## Research highlights

1. MiR-337-5p knockdown inhibited the progression of cardiac hypertrophy
2. MiR-337-5p targets UBQLN1 directly in cardiomyocytes
3. MiR-337-5p regulate the mTOR/70S6K signaling
